# Copy number variations independently induce autism spectrum disorder

**DOI:** 10.1042/BSR20160570

**Published:** 2017-07-07

**Authors:** Xie Yingjun, Yuan Haiming, Wang Mingbang, Zhong Liangying, Zhou Jiaxiu, Song Bing, Yin Qibin, Sun Xiaofang

**Affiliations:** 1 Key Laboratory for Major Obstetric Diseases of Guangdong Province, Key Laboratory of Reproduction and Genetics of Guangdong Higher Education Institutes, The Third Affiliated Hospital of Guangzhou Medical University, Guangzhou 510150, Guangdong, PR China; 2 Guangzhou Kingmed Center for Clinical Laboratory Co., Ltd., Guangzhou 510330, Guangdong, PR China; 3 KingMed School of Laboratory Medicine, Guangzhou Medical University, Guangzhou 510330, Guangdong, PR China; 4 Shenzhen Following Precision Medical Research Institute, Shenzhen 518000, Guangdong, China; 5 ImunoBio Co., Ltd., Shenzhen 518000, Guangdong, China; 6 Key Laboratory of Birth Defects, Children’s Hospital of Fudan University, Shanghai 201102, China; 7 Department of Laboratory Medicine, The First Affiliated Hospital of Sun Yat-sen University, Guangzhou 510080, Guangdong, PR China; 8 Division of Psychology, Shenzhen Children’s Hospital, Shenzhen, Guangdong, China; 9 Northeast Yucai School, Shenyang 110179, Liaoning, PR China

**Keywords:** Autism spectrum disorders, Copy number variation, Enrichment Analysis, Gene, Syndrome

## Abstract

The examination of copy number variation (CNV) is critical to understand the etiology of the CNV-related autism spectrum disorders (ASD). DNA samples were obtained from 64 ASD probands, which were genotyped on an Affymetrix CytoScan HD platform. qPCR or FISH were used as a validation for some novel recurrent CNVs. We further compared the clinical phenotypes of the genes in the Database of Chromosomal Imbalance and Phenotype in Humans Using Ensembl Resources (DECIPHER) database with these overlapping genes. Using vast, readily available databases with previously reported clinically relevant CNVs from human populations, the genes were evaluated using Enrichment Analysis and GO Slim Classification. By using the Ploysearch2 software, we identified the interaction relationship between significant genes and known ASD genes. A total of 29 CNVs, overlapping with 520 genes, including 315 OMIM genes, were identified. Additionally, myocyte enhancer factor 2 family (MEF2C) with two cases of CNV overlapping were also identified. Enrichment analysis showed that the 520 genes are most likely to be related to membrane components with protein-binding functions involved in metabolic processes. In the interaction network of those genes, the known ASD genes are mostly at the core position and the significant genes found in our samples are closely related to the known ASD genes. CNVs should be an independent factor to induce autism. With the strategy of our study, we could find the ASDs candidate genes by CNV data and review certain pathogenesis of this disorder. Those CNVs were associated with ASD and they may contribute to ASD by affecting the ASD-related genes.

## Introduction

ASDs (OMIM 209850) represent a group of neurodevelopmental disorders present in 1% of the population, characterized by impairments in communication and reciprocal social interactions [1]. Approximately 10% of the ASD population possesses large chromosomal rearrangements [1,2]. In recent years, chromosomal microarray analyses (CMA) have offered high diagnostic ability for the detection of genomic CNVs in clinical diagnostics. While whole-exome and whole-genome technologies identify interesting single nucleotide variants and show promise in detecting in/dels and copy number changes in ASDs, the genetics of ASDs are heterogeneous and not fully understood [2,3]. CNVs alter the genome structure leading to Mendelian diseases and complex traits, including ASDs. The contribution of CNVs to genomic disorders is not only via *de novo* occurrence, X-linked and recessive inheritance but also through mosaicism, imprinting, digenic inheritance and gene copy number dose dependent effects [4]. Thus, it is be important to relate the genes affected with CNVs to clinical and functional phenotypic features.

Several CNV studies in autism have identified associated genes and loci in European individuals and Han Chinese population controls [5–8]. Genetic studies on ASD in Han Chinese individuals have primarily been presented as case reports or association studies of particular common single nucleotide polymorphisms in ASD populations of European ancestry [9]. However, in the present study, we identified autism-associated genes from CNVs in 64 ASD samples and databases, and conducted additional analyses of these genes overlapping with enrichment analysis to further improve the results obtained from previous studies [5–8].

## Experimental procedures

### Sample selection

A total of 64 ASD-affected individuals and their families were referred to the Clinical Genetics Service for genetic testing. The probands diagnosis and study inclusion criteria were completed as previously described [9]. The Autism Behavior Checklist (ABC) and Childhood Autism Rating Scale (CARS) were used for the diagnosis. We assessed ASD probands with standardized measures of intelligence, language, and adaptive function and collected information on developmental, medical, and physical measures and family history (Supplementary material). All data were collected with the informed consent of the patients. Ethical approval for the present study was obtained from the hospital.

#### Consent for publication

The consent to publish has been obtained from the guardians of all the involved children.

#### Ethical approval

Ethical approval for the present study was obtained from the Ethics Committee of the Third Affiliated Hospital of Guangzhou Medical University.

### Genotyping and variant identification

DNA was isolated from 64 samples with ASD using the QIAamp DNA Mini Kit (Qiagen Benelux B.V., Venlo, Netherlands). Genotyping was performed on the Affymetrix CytoScanHD platform (Santa Clara, CA, U.S.A.) according to the manufacturer’s instructions. The ChAS software package (Santa Clara, CA, U.S.A.) was used for all the analyses. The cutoffs for the detection criteria for CNVs were set at 200 kb for gains, 100 kb for losses and 10000 kb for Regions of Homozygosity(ROH).

All observed copy number changes were compared with the CNVs annotated in the Database of Genomic Variants (DGV; http://projects.tcag.ca/variation/) and the UCSC genome browser (http://genome.ucsc.edu/). The gene content of CNVs of interest were determined using the UCSC Browser based on GRCH37. CNVs located in segmental duplications and repetitive regions were removed, and CNVs overlapping with the in-house benign CNV database were also removed. Each of the CNVs were further evaluated with respect to the affected genes likely to be associated with ASD phenotypic features observed in the patients.

### CNV verification and representation

Two independent methods were used for verifying the accuracy of our CNV algorithm. First, FISH was used when once the novel recurrent CNVs were detected, some of the results had already been published [10]. Second, 20 CNV regions at different sizes were randomly selected and qPCR technology was used for detection. Each PCR detection system was repeated three times and the corresponding control groups were set. Compared with the control region, in the detection regions, only the copy number greater than 1.4 times or less than 0.7 times, could be considered as copy number gain (gene duplication) or copy number loss (gene deletion). In addition, S.D. of the multiple must be less than 1 to assure the reliability of the experiment.

### Database mining

In addition, the intersecting CNV regions were extracted as relatively reliable CNVs associated with autism. The CNVs were further analyzed for the functional annotation of genes, transcripts, and drugs and disease relationships, and the relationship between autism and this information was further analyzed. We focused on the affected genes, including encoding and non-coding genes. The genes identified in the database were defined as having suspected gene associations with autism. We further compared the clinical phenotypes of the genes in the Database of Chromosomal Imbalance and Phenotype in Humans Using Ensembl Resources (DECIPHER) database with these overlapping genes.

### Functional analysis

The bioinformatics analysis for gene functional analysis was performed using WebGestalt (http://bioinfo.vanderbilt.edu/webgestalt/) [11]. Moreover, we also analyzed the relation of enriched GO item and the associated genes between them.

### Comparison with other similar studies

In order to better study the CNVs found in our study, we also made a comparison with the database. We extracted the CNV regions that contain the ASD-related genes from the clinical variation achieved in the dbVar database (https://www.ncbi.nlm.nih.gov/dbvar) of NCBI and downloaded the ASD-related CNV regions reported in the autism databases, SFARI gene database (https://gene.sfari.org/autdb) and National Database for Autism Research (NDAR) database (https://ndar.nih.gov/).

In order to further investigate the relation between those genes and ASD, we first collected the genes associated with ASD reported in the literatures by using the Ploysearch2 software (https://ploysearch.cs.ualberta.ca/) and then identified the interaction/relationship between significant genes and known genes.

### Availability of supporting data

Affymetrix cytoscan HD (http://media.affymetrix.com/support/technical/datasheets/cytoscan_hd_datasheet.pdf).

Chromosome Analysis Suite Software, Version 3.1 (http://www.affymetrix.com/support/technical/software_downloads.affx).

## Results

Amongst a cohort of ASD patients, SNP array identified 29 (45%, 29/64) CNVs: 9.3% of probands (6/64) carried a recurrent microdeletion/duplication syndrome (Table 1); and 19 non-recurrent CNVs (Table 2). Additionally, *MEF2C* with two cases of CNVs overlap were also identified (Table 3). These CNVs overlapped with 520 genes, including 315 OMIM genes, present on chromosomes 2, 4, 5, 7, 8, 12, 14, 15, 16, and 22. We compared these 520 genes using WebGestalt (total number of user IDs: 520). A total of 496 user IDs were unambiguously mapped to 487 unique Entrez Gene IDs, and 24 user IDs were mapped to multiple Entrez Gene IDs or could not be mapped to any Entrez Gene ID. Thus, the Enrichment Analysis and GO Slim Classification was based on the 487 unique Entrez Gene IDs. The results of the molecular functional classification, showing each biological process and cellular component category, are presented in Table 4.

**Table 1:** Recurrent CNVs in ASDs

Sample ID	Size (kbp)	Gene count	OMIM® genes count	Microarray nomenclature	Syndrome overlap
**1471**	11269.38	93	55	arr[hg19] 3q27.2q29(184,522,306-195,791,682)×1	3q29 microdeletion syndrome
**7714**	2248.396	34	18	arr[hg19] 5p15.33(113,576-2,361,972)×1	Cri du chat syndrome
	10854.223	122	74	arr[hg19] 16q23.2(79,281,580-90,155,062)×3	
**7756**	1421.098	27	23	arr[hg19] 7q11.23(72,725,760-74,146,858)×3	7q11.23 duplication syndrome
**4876**	232.163	12	9	arr[hg19] 16p11.2(28,819,028-29,051,191)×1	16p11.2-p12.2 microdeletion syndrome
**7687**	577.588	29	18	arr[hg19] 16p11.2(29,567,295-30,144,883)×1	16p11.2-p12.2 microdeletion syndrome
**2543**	9079.75	131	76	arr[hg19] 22q13.2q13.33(42,118,088-51,197,838)×1	22q13 deletion syndrome
**4229**	903.193	35	26	arr[hg19] 22q13.33(50,294,532–51,197,725)×1	22q13 deletion syndrome

**Table 2:** Non-recurrent CNVs in ASDs

Sample ID	Size (kbp)	Microarray nomenclature	Genes
**1033**	211.662	arr[hg19] 2q36.3(230,659,011-230,870,673)×3	TRIP12*, FBXO36*
**7817**	550.981	arr[hg19] 2q37.3(240,739,224-241,290,205)×3	MIR4786, NDUFA10*, OR6B2, PRR21, OR6B3, MYEOV2, OTOS*
**9266**	233.526	arr[hg19] 3q28(188,332,838-188,566,364)×1	LPP*
**7824**	369.331	arr[hg19] 4q24(107,035,056-107,404,387)×1	TBCK, AIMP1*, GIMD1
**7857**	376.335	arr[hg19] 4q35.2(189,007,828-189,384,163)×3	TRIML2, TRIML1, LOC401164
**3101**	176.934	arr[hg19] 5q14.3(88,132,559-88,309,493)×1	MEF2C*
**7857**	2289.57	arr[hg19] 5q14.3(88,196,115-90,485,685)×1	MEF2C*, MIR3660, CETN3*, MBLAC2, POLR3G, LYSMD3, GPR98*
**3322**	896.359	arr[hg19] 8q23.3(116,237,764-117,134,123)×1	TRPS1*, LINC00536
**7032**	386.355	arr[hg19] 8p22(17,371,318-17,757,673)×1	SLC7A2*, PDGFRL*, MTUS1*, FGL1*
**8690**	151.812	arr[hg19] 12q13.11(47,139,554-47,291,366)×1	SLC38A4*
**4211**	252.233	arr[hg19] 14q13.1(33,428,360-33,680,593)×1	NPAS3*
**1248**	440.507	arr[hg19] 15q13.3(32,003,537-32,444,044)×3	CHRNA7*
**4626**	126.31	arr[hg19] 15q15.3(43,907,775-44,034,085)×1	STRC*, CATSPER2*, CKMT1A*, CATSPER2P1
**5977**	142.21	arr[hg19] 15q11.2(22,770,421-22,912,631)×1	TUBGCP5*, CYFIP1*
**5977**	274.255	arr[hg19] 15q11.2(22,917,396-23,191,651)×1	CYFIP1*, NIPA2*, NIPA1*, LOC283683, WHAMMP3
**7756**	165.56	arr[hg19] 15q15.3(43,889,174-44,054,734)×1	RNU6-28P, CKMT1B*, STRC*, CATSPER2*, CKMT1A8, CATSPER2P1, PDIA3*
**9943**	143.975	arr[hg19] 16p12.2(21,596,299-21,740,274)×1	METTL9*, IGSF6*, OTOA*
**7769**	575.16	arr[hg19] 16q23.1(78,434,692-79,009,852)×3	WWOX*
**7769**	281.388	arr[hg19] 16q23.1q23.2(79,191,466-79,472,854)×3	WWOX*
**9266**	252.225	arr[hg19] 18q22.2(68,060,722-68,312,947)×3	GTSCR1

*OMIM genes

**Table 3:** The character of genes with two cases overlap

Gene	Case ID	Loss/gain	Location [hg19]	Function	OMIM	HI score	DDG2P	Phenotype of decipher cases
**LPP**	9266,1471	Loss	3:187871072-188608460	LIM domain containing preferred translocation partner in lipoma	+	4.34	_	+
**MEF2C**	3101, 7857	Loss	5:88013975-88199922	Myocyte enhancer factor 2C	+	0.26	+	+
**CHRNA7**	1248, 0842	Gain	15:32322691-32464722	Cholinergic receptor, nicotinic, α 7 (neuronal)	+	40.52	_	+

DDG2P, the Developmental Disorders Genotype-Phenotype Database; HI, haploinsufficiency.

**Table 4.** Genes of functional classification by using WebGestalt

Function	Gene ratio (total gene 487)
**Moleclular function categories**	
** Protein binding**	166/487
** Lon binding**	116/487
** Nucleic acid binding**	61/487
** Nucleic binding**	54/487
** Hydrolase activity**	47/487
**Biological process categories**	
** Metabolic process**	196/487
** Biological regulation**	168/487
** Response to stimulus**	141/487
** Multicellular organismal process**	122/487
**Developmental process**	98/487
** Cellular component categories**	
** Membrane**	155/487
** Nucleus**	106/487
** Macromolecular comples**	75/487
** Membrane-enclosed lumen**	66/487
** Cytosol**	44/487

Comparing the CNV regions with the CNVs in the above databases (dbVar database, FARI gene database, NDAR database), we found 472 (84.1% of total) CNV regions overlapping with those in the databases (Figure 1). There are 89 CNV regions that do not overlap with the databases. In addition, we compared the CNVs in our ASD samples with CNVs in the normal individuals and identified the CNVs in our ASD samples showing significantly different from those of normal individuals. Then we compared them with those in the databases. At this time, there were 72 CNVs (87.8% of the total) overlapping with the databases and there were 10 CNVs not overlapping with databases.

**Figure 1:** Number of overlapped CNV regions with Sfari, ClinVar and NDAD

As those genes show significantly different CNVs amongst ASD patients and normal controls, they are related with the ASD. In the interaction network of those genes, the known ASD genes are mostly at the core position and the significant genes found in our samples are closely related to the known genes. Amongst the significant genes, *MAPK11, TSC2*, and *F10* are also at the core position (Figure 2).

**Figure 2:** Interaction network of our CNVs genes

## Discussion

In the present study, we used a conceptually different approach, evaluating CNV hotspots across 64 ASD samples to analyze the human genome using vast, readily available databases with previously reported clinically relevant CNVs from human populations, thereby enhancing the current understanding of the etiology of CNVs in ASDs. Several microdeletion/microduplication syndromes detected through CMA have shown symptoms including ASD and comparison of the data with other ASD database found that 472 (84.1% of total) CNV regions overlap with these databases. Thus, the results of the present study are consistent with previous studies showing that CNVs are one of the multiple factors contributing to the development of an ASD phenotype [7].

In the present study, one autism-related CNV deletion gene was identified : *MEF2C* (Table 3). In particular, *MEF2C* exhibited a high HI score (e.g., 0–10%), indicating that these genes have a higher likelihood of exhibiting HI, with the most obvious pathogenic mechanism being heterozygous loss-of-function mutations (such as large, rare deletions) where a functional copy of a gene is insufficient to maintain the normal function [12]. As it was known that the transcription factors of the myocyte enhancer factor 2 family (MEF2 A–D) are highly expressed in the brain and play a key role in neuronal survival/apoptosis, differentiation and synaptic plasticity [13]. Previous study also showed that *MEF2C* limits excessive synapse formation during activity-dependent refinement of synaptic connectivity and thus facilitates hippocampal-dependent learning and memory [14]. In fact, increasing evidence has demonstrated the relevance of synapse dysfunction as a major determinant in many neurological diseases including autism [15]. Thus, the results of the present study provided evidence that the MEF2C deletion might be a factor for the induction of autism.

Recent studies have identified more than 103 genes and 44 genomic loci with mutations among individuals with some form of ASD [16]. The CNV-contained genes found in our study, *MAPK11, TSC2*, and *F10* are the known ASD-associated genes, which locate at the core position of interaction network, indicating that those CNVs were associated with ASD and they may contribute to ASD by affecting the ASD-related genes. In the present study, enrichment analysis showed that the 520 genes are most likely to be associated with membrane components with protein-binding functions involving metabolic processes, reflecting the tardive dyskinesia in autism and providing the biological basis of autism susceptibility. Based on the previous study, several metabolic defects have been associated with autistic symptoms with a rate higher than that found in the general population, and, inborn errors of metabolism (IEM) can probably account for less than 5% of individuals [17]. In addition, inherited metabolic disorders (IMD) responsible for ASDs are usually identified via clinical manifestations such as microcephaly, dysmorphic features, convulsions, and hepatosplenomegaly, and, patients with no additional clinical symptoms suggestive of an IMD may be diagnosed as having an idiopathic ASD [18,19]. Indeed, genetic factors leading to the abnormal expression of nerve growth associated proteins, enzymes, receptors, and neurotransmitters result in the abnormal proliferation and differentiation of neurones, including excessive trim, abnormal synaptic connections, and abnormal neural circuits [20–23]. As a result, it is logical that genes with associated metabolic disorders may also be considered as candidate ASDs’ genes.

In addition, genome variations are one of the genetic etiology of human disease. In the field of autism, point mutation is the top priority in the researches related with pathological genetic characteristics [24–26]. Several human syndromes derived from a single gene mutation increase the risk for ASD: such as fragile X-chromosome syndrome and Timothy syndrome [27,28]. Except for CNVs, CMA platform cannot detect other genome variations, such as point mutation, which could at least explain the patients without CNVs in our study.

## Conclusion

The investigation of the CNVs associated with ASD is promising for deciphering the genetic effects of these diseases. With the strategy of our study by genotyping 64 ASD patients, the results suggest that CNVs are one of the multiple factors contributing to the development of an ASD. The pathogenesis at least includes: (i) genes with metabolic disorders associated may be considered as candidate ASDs genes; (ii) CNV contains genes are functionally and closely related to the known ASDs genes. These results also reveal a significant gap in the function of non-coding genes for autism, which should be analyzed in follow-up studies. As microarrays remain the gold standard for CNV detection, further studies on CNVs to identify new genes that might contribute to ASDs will continue.

### Summary of findings

- Copy number variations (CNVs) are one of the multiple factors contributing to the development of an autism spectrum disorder (ASD) phenotype.
- The myocyte enhancer factor 2 family (MEF2C) deletion might be a factor in the induction of autism.
- Genes associated with metabolic disorders may also be considered as candidate ASD genes.
- ASD genes found in our samples are closely related to the known ASD genes.

## Abbreviations

ASD: autism spectrum disorder
CNV: copy number variation
CMA: chromosomal microarray analysis
GO: Gene Ontology
HI: haploinsufficiency
IEM: inborn errors of metabolism
IMD: inherited metabolic disorder
MEF2: myocyte enhancer factor 2 family
NDAD: National Database for Autism Research
qPCR: quantitative polymerase chain reaction
S.D.: standard deviation
SNP: single nucleotide polymorphism
